The article "Helicobacter pylori promotes inflammatory factor secretion and lung injury through VacA exotoxin-mediated activation of NF-κB signaling" was retracted in 2026. Reasons: concerns about the data; concerns about the results or conclusions.

# Helicobacter pylori *promotes inflammatory factor secretion and lung injury through VacA exotoxin-mediated activation of NF-κB signaling*

**DOI:** 10.1080/21655979.2022.2071011

**Published:** 2022-05-21

**Authors:** Meizhu Chen, Xueping Huang, Minzhao Gao, Zhipeng Yang, Zhaoxiong Fang, Jinqi Wei, Baihe Wu

**Affiliations:** a Department of Pulmonary and Critical Care Medicine (PCCM), The Fifth Affiliated Hospital of Sun Yat-sen University, Zhuhai, China; b Department of Gastroenterology, Fujian Provincial Hospital, Fuzhou, China; c Department of Gastroenterology, Shengli Clinical Medical College of Fujian Medical University, Fuzhou, China; d Department of Gastroenterology, The Fifth Affiliated Hospital of Sun Yat-sen University, Zhuhai, China; e Department of Gastroenterology, Dongguan Tungwah Hospital, DongGuan, China

**Keywords:** Helicobacter pylori, VacA, inflammatory cytokines, endothelial dysfunction, NF-κB signaling

## Abstract

Previous reports have shown that *Helicobacter pylori* (*H. pylori*) infection is associated with respiratory diseases. However, the pathogenesis remains unclear. Vacuolating cytotoxin A (VacA) is a major *H. pylori* exotoxin. In this study, we investigated the signaling pathways involved in the inflammatory response to *H. pylori* infection and VacA. Mice were treated with *H. pylori* and VacA, and histopathological analysis of lung tissues was performed using hematoxylin-eosin, Masson’s trichrome, and periodic acid Schiff staining. The secretion of inflammatory cytokines was evaluated by enzyme-linked immunosorbent assay. The expression of VacA, nuclear factor-kappa B (NF-κB), and p65 NF-κB was analyzed by Western blotting and immunofluorescence. Cell proliferation and apoptosis were assessed using the MTS assay and flow cytometry, respectively. In mice, *H. pylori* infection and VacA treatment promoted the secretion of the inflammatory factors interleukin 1β (IL-1β), tumor necrosis factor α (TNF-α), IL-6, and IL-8, increased p65 NF-κB protein phosphorylation, and induced lung injury. Furthermore, *H. pylori* infection promoted VacA production. In an *in vitro* cell model, VacA treatment significantly suppressed the proliferation of WI-38 and BEAS-2B cells, promoted apoptosis, induced TNF-α, IL-1β, IL-6, and IL-8 secretion, and promoted p65 NF-κB protein phosphorylation and NF-κB nuclear transfer. The NF-κB inhibitor BAY11-7082 alleviated VacA-induced inflammation and apoptosis and increased cell viability. In conclusion, VacA promotes the secretion of inflammatory factors and induces lung injury through NF-κB signaling.

## Highlights

- *H. pylori* infection and VacA treatment enhanced lung injury in mice.
- *H. pylori* infection promotes VacA production in mice.
- VacA treatment promotes the secretion of the inflammatory factors.
- VacA treatment activates NF-κB pathway.

## Introduction

*Helicobacter pylori* (*H. pylori*) infection is closely associated with various human gastric diseases, such as gastritis, gastric ulcers, gastric atrophy, and gastric cancer [1–3]. Approximately half of the global population is infected with *H. pylori*, resulting in high mortality [4]. Recently, *H. pylori* infection was found to be related to extra-digestive diseases, such as autoimmune, respiratory, and cardiovascular diseases [5,6]. Inflammation caused by *H. pylori* infection is considered the main cause of these diseases [7]; Arismendi et al. reported that *H. pylori* infection leads to lung injury by recruiting inflammatory cells and promoting the secretion of inflammatory cytokines, which induces morphological changes in the lung tissue [8]. However, the mechanisms by which *H. pylori* infection causes respiratory diseases remain unclear. Vacuolating cytotoxin A (VacA), a major exotoxin of *H. pylori*, can induce vacuolation, inhibit T cell function, regulate autophagy, and promote cell death [9,10]. Recently, Nakashima et al [11]. found that VacA promotes the secretion of interleukin-8 (IL-8) and interleukin-6 (IL-6), potentially inducing respiratory diseases. Therefore, VacA may be the main factor in *H. pylori-*mediated respiratory diseases.

*H. pylori* infection induced lung injury via increasing the expression of inflammatory mediators using a mouse model [8]. *H. pylori* stimulates immune response and long-term inflammation which may be one of the causes of lung injury in the human body [12]. *H. pylori* infection activated NF-κB signaling pathway leading to the deleterious gastric pathophysiology and gastric diseases [13]. The nuclear factor-kappa B (NF-κB) pathway is closely associated with inflammatory cytokine secretion, which has a positive feedback–based regulatory relationship with inflammatory factors such as interleukin 1β (IL-1β) and tumor necrosis factor α (TNF-α) [14]. VacA promoted inflammatory cytokine secretion and cell apoptosis in human monocytic cell line via the activation of NF-κB [15]. These studies have shown that *H. pylori* infection and VacA treatment can activate the NF-κB signaling pathway to promote the expression and secretion of inflammatory factors. However, whether *H. pylori* infection and VacA treatment causes lung injury via the NF-κB pathway remains unknown.

This study hypothesized that VacA, a major *H. pylori* exotoxin, promote inflammatory cytokine secretion and lung lung injury via regulating NF-κB signaling pathway. In this study, we investigated the pulmonary effects of *H. pylori* infection and VacA treatment in mice and evaluated the molecular mechanisms of the NF-κB signaling pathway. In addition, we verified the injury-inducing effect and mechanism of action of VacA *in vitro* in WI-38 and BEAS-2B cells. By clarifying the mechanism of *H. pylori* infection, this study may provide a foundation for identifying novel therapeutic targets.

## Methods

### Animals

Male BALB/c wild-type (WT) mice (6–12 weeks old), weighing approximately 25–30 g, were obtained from the Medical Experimental Animal Center of the Laboratory Animal Management Center of Southern Medical University. The mice had free access to sterile food and water during the entire experimental period and were maintained under a 12 h/12 h light/dark cycle at 25°C. All animal experiments were approved by the Fifth Affiliated Hospital of Sun Yat-sen University (Approval time: 23 March 2021).

### *Bacteria*, H. pylori *infection, and VacA treatment*

*H. pylori* strain NCTC 11638 (National Institute for Communicable Disease Control and Prevention, Chinese Center for Disease Control and Prevention, Beijing, China) was grown and prepared as described previously [8]. Briefly, 2 × 10^8^ CFU/mL of bacterial suspension was used to infect the mice. VacA (recombinant VacA protein, *H. pylori* A210016, Baiaolaibo, Beijing, China) was dissolved in phosphate buffered saline (PBS). Mice were divided into four groups of six: normal, *H. pylori-*infected, negative control (NC), and VacA-treated. In the normal group, the mice received no treatment. In the *H. pylori*-infected group, 50 μL of bacterial suspension was administered by orotracheal instillation once a day for 3 d. In the VacA-treated group, 10 mg/mL of VacA was administered by orotracheal instillation once a day for 3 d. In the NC group, an equal amount of sterile 1× PBS (pH 7.4) was administered once a day for 3 d. After 14 d, the mice were sacrificed. Blood samples were collected for cytokine analysis, and lung tissue samples were quickly harvested and snap frozen in liquid nitrogen until analysis.

### Histopathological analysis of lung tissues

Hematoxylin-eosin (H&E), Masson’s trichrome, and periodic acid Schiff (PAS) staining kits were obtained from Solarbio Life Science (Beijing, China) [16]. Harvested lung tissue samples were fixed and mounted. Sections were then stained, and histopathological analysis was performed using light microscopy (Olympus, Tokyo, Japan). Five fields per sample were analyzed.

### Immunofluorescence assay

For the immunofluorescence assay, sections of lung tissue were incubated first with anti-p65 NF-κB antibody (Abcam, Cambridge, MA, USA; 1:100) and then with secondary antibody (Abcam; 1:3000) at 37°C for 1 h, after which they were counterstained with DAPI [17]. Samples were observed under a fluorescence microscope (Olympus CX23, Tokyo, Japan).

### Western blotting

For Western blotting, total protein was separated by 10% sodium dodecyl sulfate polyacrylamide gel electrophoresis and transferred to polyvinylidene difluoride membranes (Millipore, Atlanta, GA, USA) [17]. After washing and blocking, the membranes were incubated with primary antibodies against VacA (sc-32,746, Santa Cruz Biotechnology, Santa Cruz, CA, USA, 1:500), p65 NF-κB (ab32536, 1:5000), p-p65 NF-κB (ab76302, 1:1000), and GAPDH (ab8245; Abcam, 1:10,000). After washing again, the membranes were incubated with secondary antibody (ab205718 and ab6728; Abcam, 1:10,000) for 2 h at 25°C. Protein bands were detected using an enhanced chemiluminescence kit (Pierce, Rockford, IL, USA).

### RT-qPCR

For RT-qPCR, the relative expression level of CNN3 was calculated using the 2^–ΔΔCT^ method [18]. The expression of TNF-α, IL-1β, IL-6, and IL-8 was measured by qRT-PCR using SYBR GREEN qPCR Super Mix (Invitrogen). Primers as follows: GAPDH: 5’-GCTCATTTGCAGGGGGGAG-3’ and 5’-GTTGGTGGTGCAGGAGGCA-3’; IL-1β: 5’-CTTGGTGATGTCTGGTCCAT-3’ and 5’-CCTTGTACAAAGGACATGGAG-3’; IL-6: 5’-CCAGAGCTGTGCAGATGAGT-3’ and 5’-CTGCAGCTTCGTCAGCAGGC-3’; IL-8: 5’-AGTGCATAAAGACATACTCC-3’ and 5’-GCTTTACAATAATTTCTGTG-3’; and TNF-a: 5’-CAGTCAGATCATCTTCTCGA-3’ and 5’-CCGGCGGTTCAGCCACTGGA-3’.

### Luciferase activity assay

The procedure of Luciferase activity assay is shown in previous studies [19]. Briefly, WI-38 and BEAS-2B cells were transiently co-transfected with NF-κB reporter and TK Renilla lucifer-ase plasmids using Lipofectamine™ 2000 (Invitrogen). After culture 24 h, the luciferase activity of the supernatant was detected using a Dual-luciferase reporter assay system, and relative fluorescence reporter activity were designated as the activity of firefly luciferase normalized to that of Renilla luciferase.

### ELISA

TNF-α, IL-1β, IL-6, and IL-8 levels in blood samples and cell culture supernatants were measured using ELISA. All ELISA kits were purchased from Bioss (Beijing, China).

### Cell treatment

WI-38 and BEAS-2B cells were cultured in 6-well plates at a density of 1.0 × 10^5^ cells per well. The cells were divided into three groups: normal, VacA-treated, and negative control (NC). In the normal group, cells were cultured normally. In the VacA-treated group, 1 μg/mL VacA (final concentration) was added to the medium. In the NC group, an equal amount of PBS was added to the medium. Next, the NF-κB inhibitor BAY11-7082 was used to investigate the relationship between VacA and NF-κB. In the VacA + inhibitor group, 1 μg/mL VacA and 5 μmol/L BAY11-7082 (final concentration) were added to the medium. In the VacA + PBS group, VacA (1 μg/mL) and PBS were added to the medium. After 48 h of incubation, the cells and culture supernatants were collected by centrifugation. Three independent experiments were performed.

### Cell proliferation and apoptosis assays

After treatment, the CellTiter 96® AQ_ueous_ One Solution Cell Proliferation Assay kit (MTS assay; Promega, Madison, WI, USA) was used to evaluate cell proliferation. Cells were double-stained using the Annexin V-FITC Apoptosis Detection Kit (Keygentec, Nanjing, China), following the manufacturer’s instructions. The percentage of apoptotic cells was assessed by NovoCyte 4025 flow cytometry and NovoExpress software analysis (ACEA Biosciences, Agilent, Hangzhou, China). The original images of apoptosis were shown in Supplementary 4_flow apoptosis pictures.

### Statistical analysis

Statistical analysis was performed using SPSS 22.0 statistical software (IBM Corp., Armonk, NY, USA). All data conformed to a normal distribution and are expressed as the mean ± standard deviation (SD). Differences among the normal, *H. pylori-*infected, NC, and VacA-treated groups were analyzed using Student’s *t*-test. Comparisons among the normal, NC, and VacA-treated groups and among the VacA, VacA + PBS, and VacA + inhibitor groups were performed using one-way analysis of variance (ANOVA) followed by Dunnett’s test. Statistical significance was set at *P < *0.05.

## Results

### Histopathological analysis of lung tissues

To study the pulmonary effect of *H. pylori* infection and VacA treatment in mice, histological analysis of lung tissues was performed using H&E, Masson’s trichrome, and PAS staining. H&E staining indicated significant alveolar hemorrhage, inflammatory cell infiltration, and alveolar fusion in the pulmonary tissue of the *H. pylori*-infected group, compared to that of the normal group. Masson’s staining produced blue-colored connective tissues in the *H. pylori-*infected group, indicating obvious fibrosis in the pulmonary tissue. PAS staining revealed the presence of macrophages in lung tissue in the *H. pylori*-infected group (Figure 1). The NC group exhibited results similar to those of the normal group and the VacA-treated group exhibited results similar to those of the *H. pylori*-infected group (Figure 1).

**Figure 1.** Effect of *H. pylori* infection and VacA treatment on mouse lung tissue, examined using hematoxylin-eosin (H&E), Masson’s trichrome, and periodic acid Schiff stains. (40 ×).

### H. pylori *infection and VacA treatment promoted expression of inflammatory factors and NF-κB signaling in mice*

To determine the effect of *H. pylori* infection and VacA treatment on the expression of inflammatory factors, ELISA was used to measure the expression of TNF-α, IL-1β, IL-6, and IL-8 in the serum of mice infected with *H. pylori* and treated with VacA. Compared to the normal and NC groups, the *H. pylori*-infected group exhibited increased levels of TNF-α, IL-1β, IL-6, and IL-8; these effects were also observed in the VacA-treated group (Figure 2a). Compared to the normal and NC groups, the *H. pylori*-infected group exhibited higher levels of VacA and p-p65 NF-κB proteins, but p65 NF-κB protein levels were unaffected. Similar results were found in the VacA-treated group (Figure 2b). Immunofluorescence assay results showed that *H. pylori* infection and VacA treatment promoted the transfer of NF-KB from the cytoplasm to the nucleus (Figure 2c).

**Figure 2.** Effect of *H. pylori* infection and VacA treatment on the expression of inflammatory factors and NF-κB signaling in mice. (a) Levels of TNF-α, IL-1β, IL-6, and IL-8 in mouse blood samples after *H. pylori* infection and VacA treatment were measured by ELISA. (b) VacA, p-p65 NF-κB, and p65 NF-κB protein expression in mouse lung tissue after *H. pylori* infection and VacA treatment was analyzed by Western blotting. (c) p-p65 NF-κB protein expression in mouse lung tissue after *H. pylori* infection and VacA treatment was measured by immunofluorescence assay. Red arrows indicate the translocation of p65 NF-κB to the nucleus. (*P < 0.05).

### VacA treatment suppressed proliferation and promoted apoptosis of lung cells

To study the effect of VacA treatment on lung cell proliferation, the viability of WI-38 and BEAS-2B cells after VacA treatment for 48 h was measured via MTS assay. Compared to that in the normal and NC groups, cell viability was significantly suppressed in the VacA treatment group (Figure 3a and 3c). Moreover, VacA treatment significantly promoted apoptosis (Figure 3b and 3d).

**Figure 3.** Effect of VacA treatment on WI-38 and BEAS-2B cell viability and apoptosis. (a and c) Cell viability after VacA treatment was assessed by MTS assay. (b and d) Cell apoptosis after VacA treatment was assessed by flow cytometry. (*vs* normal, *P < 0.05, *vs* NC, *^#^P* < 0.05).

### VacA treatment promoted expression of inflammatory factors and NF-κB signaling in lung cells

To analyze the effect of VacA treatment on the expression of inflammatory factors in lung cells, the levels of TNF-α, IL-1β, IL-6, and IL-8 in the culture supernatants of VacA-treated WI-38 and BEAS-2B cells were measured by ELISA and qRT-PCR. Compared to those in the normal and NC groups, the levels of TNF-α, IL-1β, IL-6, and IL-8 were significantly increased in the VacA-treated group (Figure 4a and 4b). Compared to the normal group, the VacA-treated group exhibited significantly higher p-p65 NF-κB protein expression, whereas p65 NF-κB protein expression remained unchanged, suggesting that VacA treatment significantly enhanced the phosphorylation of p65 NF-κB protein (Figure 4c). Luciferase activity assay found that the reporter activity of NF-κB in both WI-38 and BEAS-2B cells was significantly activated after VacA treatment (Figure 4d). Additionally, immunofluorescence and western blot assay results showed that p65 NF-κB protein expression in the nucleus was obviously enhanced after VacA treatment (Figure 4e and 4f).

**Figure 4.** Effect of VacA treatment on the expression of inflammatory factors and NF-κB signaling in WI-38 and BEAS-2B cells. (a) Levels of TNF-α, IL-1β, IL-6, and IL-8 in cell supernatants after VacA treatment were measured by ELISA. (b) TNF-α, IL-1β, IL-6, and IL-8 mRNA expression in WI-38 and BEAS-2B cells after VacA treatment were measured by RT-qPCR. (c) p-p65, NF-κB, and p65 NF-κB protein expression in WI-38 and BEAS-2B cells after VacA treatment was measured by Western blotting. (d) NF- κB fluorescence intensity after VacA treatment was determined by luciferase activity assay. (e) The expression of p65 NF- κB fluorescence in nucleus and cytoplasm was analyzed by immunofluorescence. Red arrows indicate the translocation of p65 NF-κB to the nucleus. (f) The expression of p65 NF- κB fluorescence in nucleus and cytoplasm was analyzed by Western blotting. (*vs* normal, *P < 0.05, *vs* NC, *^#^P* < 0.05).

### The NF-κB signaling pathway is regulated by VacA

To determine whether NF-κB is a downstream pathway regulated by VacA, cells were incubated with both NF-κB inhibitor and VacA protein. The p-p65 NF-κB protein level was significantly reduced, whereas the p65 NF-κB protein level remained unchanged in the VacA + inhibitor group compared to that in the VacA and VacA + PBS groups (Figure 5a). Additionally, immunofluorescence and western blot assay results showed that p65 NF-κB protein expression in the nucleus was obviously reduced in the VacA + inhibitor group (Figure 5b and 5c). Compared to those in the VacA and VacA + PBS groups, the levels of TNF-α, IL-1β, IL-6, and IL-8 in the cell and culture supernatants of WI-38 and BEAS-2B cells were significantly decreased in the VacA + inhibitor group (Figure 5d and 5e). In addition, compared to that in the VacA and VacA + PBS groups, the viability of WI-38 and BEAS-2B cells in the VacA + inhibitor group was significantly enhanced, whereas apoptosis was significantly suppressed (Figure 6).

**Figure 5.** Alleviation of VacA-induced inflammation in WI-38 and BEAS-2B cells by the NF-κB inhibitor BAY11-7082. (a) Protein expression of p-p65, NF-κB, and p65 NF-κB after co-treatment with VacA and NF-κB inhibitor was measured by Western blotting. (b) The expression of p65 NF- κB fluorescence in nucleus and cytoplasm was analyzed by immunofluorescence after after co-treatment with VacA and NF-κB inhibitor. Red arrows indicate the translocation of p65 NF-κB to the nucleus. (c) The expression of p65 NF- κB fluorescence in nucleus and cytoplasm after after co-treatment with VacA and NF-κB inhibitor was analyzed by Western blotting. (d) Levels of TNF-α, IL-1β, IL-6, and IL-8 in cell supernatants after co-treatment with VacA and NF-κB inhibitor were measured by ELISA. (e) TNF-α, IL-1β, IL-6, and IL-8 mRNA expression in cell after after co-treatment with VacA and NF-κB inhibitor were measured by RT-qPCR. (*vs* VacA group, *P < 0.05, *vs* VacA + PBS group, *^#^P* < 0.05).

**Figure 6.** Alleviation of VacA-induced apoptosis and suppression of viability by the NF-κB inhibitor BAY11-7082. (a and c) Viability of WI-38 and BEAS-2B cells after VacA treatment was assessed by MTS assay. (b and d) Apoptosis of WI-38 and BEAS-2B cells after VacA treatment was assessed by flow cytometry. (*vs* VacA group, *P < 0.05, *vs* VacA + PBS group, *^#^P* < 0.05).

## Discussion

Recently, *H. pylori* infection has been associated with many extra-digestive diseases, including respiratory diseases [20,21]. In the present study, *H. pylori* infection and VacA treatment induced morphological changes and lung tissue injury in mice. *H. pylori* infection and VacA treatment also promoted the secretion of the inflammatory factors TNF-α, IL-1β, IL-6, and IL-8, in addition to increasing p65 NF-κB protein expression. In the *in vitro* lung cell model, VacA treatment significantly suppressed cell viability, promoted apoptosis, and induced TNF-α, IL-1β, IL-6, and IL-8 production. VacA treatment also significantly promoted p65 NF-κB protein expression. The NF-κB inhibitor BAY11-7082 alleviated VacA-induced inflammation and apoptosis and enhanced cell viability. These data clearly indicate that *H. pylori* VacA promotes inflammatory factor secretion and endothelial dysfunction through the NF-κB signaling pathway, resulting in lung injury.

Recently, the association between *H. pylori* infection and certain extra-gastric manifestations, such as chronic respiratory diseases, has been investigated [22–24]. *H. pylori* DNA has been found in the bronchoalveolar lavage fluid from lung cancer patients and in lung biopsy specimens, suggesting that *H. pylori* exists in lung tissues [25]. *H. pylori* infection enhances the mRNA expression of TNF-α, IL-1β, MMP9, I-CAM, V-CAM, and IL-8 in lung tissues and promotes lung injury [8]. Similarly, we found that the lung samples from *H. pylori*-infected mice featured morphological changes and injury, and the same effects were observed following VacA treatment. These result suggest that VacA is a major H. pylori virulence factor in lung injury. Previous study found that cag-pathogenicity Island is an established H. pylori virulence factor which can enhance inflammatory response and promote gastric cancer [26], suggest that different virulence factors play a key role in different diseases. Furthermore, *H. pylori* infection enhanced VacA production in mice with lung injury, suggesting that *H. pylori* infection may cause damage via the VacA protein. *H. pylori* infection and VacA treatment also promoted the secretion of the inflammatory factors TNF-α, IL-1β, IL-6, and IL-8 in mouse serum. Subsequently, the mechanism of VacA-mediated injury was verified *in vitro* in WI-38 and BEAS-2B cells. The viability and apoptosis rate of human bronchial epithelial cells are important indicators of lung cell function. We found that infection significantly suppressed the viability of lung cells and promoted apoptosis, indicating that VacA treatment leads to bronchial epithelial cell dysfunction. Nakashima et al. reported that VacA treatment promotes IL-6 and IL-8 secretion in lung cells, leading to respiratory diseases in predisposed individuals [11]. Similarly, we found that VacA treatment induced TNF-α, IL-1β, IL-6, and IL-8 production in WI-38 and BEAS-2B cells, supporting the hypothesis that the lung epithelium is responsive to pathogenic factors of *H. pylori*.

The NF-κB pathway has been associated with severe inflammatory diseases [27,28]. We found that *H. pylori* infection and VacA treatment promoted p65 NF-κB protein phosphorylation and NF-κB nuclear transfer. These results suggest that NF-κB signaling may play a vital role in the inflammatory response and lung injury induced by *H. pylori* infection in mice. Furthermore, these findings indicate that *H. pylori* infection promotes inflammatory factor secretion, activates NF-κB signaling, and induces lung injury via the VacA exotoxin.VacA treatment significantly promoted p65 NF-κB protein phosphorylation and NF-κB nuclear transfer in WI-38 and BEAS-2B cells. The NF-κB inhibitor BAY11-7082 alleviated VacA-induced inflammation and apoptosis and enhanced cell viability. Therefore, the VacA exotoxin may promote inflammatory secretion and cell apoptosis and inhibit cell viability by activating NF-κB signaling. Combined with the results of the animal experiments, we concluded that VacA is a functional *H. pylori* protein that activates the NF-κB signaling pathway, promoting the secretion of inflammatory factors and thereby inhibiting the survival of lung cells. Previous study found that VacA secreted by *H. pylori* was recognized as pattern-recognition receptors by the toll-like receptors, NOD-like receptors, RIG-I like receptors, and C-type lectin receptors [29]. Then it can promote inflammatory cytokine secretion and cell apoptosis via activating TRAF6/IRAK4/IκBα/NF-κB pathway and promoting NF-κB nuclear transfer [29,30]. It may be the mechanism by which VacA activates NF-KB to promote the secretion of inflammatory factors in lung cells. However, this mechanism needs to be further proved. In addition, studies have shown that VacA can also regulate mitogen-activated protein kinase pathway, phosphorylation of protein kinase B pathway, and autophagy, which also had relationship with inflammation and cell apoptosis [31–33]. Therefore, whether VacA can regulate other signaling pathways in lung injury remains to be further investigated.

## Conclusion

*H. pylori* infection promotes inflammatory factor secretion and induces lung injury through the VacA exotoxin, which activates NF-κB signaling. VacA is the main mediator of respiratory diseases caused by *H. pylori* and represents a potential therapeutic target.

## Supplementary Material

Supplemental Material

## Data Availability

All date from this study are available in this published article.
